# Analysis of the Therapeutic Effect of Changyanning on Intestinal Flora in Inflammatory Bowel Disease

**DOI:** 10.1155/2022/3757763

**Published:** 2022-06-22

**Authors:** Xinyu Hu, Fuyuan Yang

**Affiliations:** Yangtze University Health Science Center, Jingzhou 434020, China

## Abstract

*Research Purposes*. Inflammatory bowel disease (IBD) is an autoimmune disease coinduced by genes, environment, and immune response, mainly including ulcerative colitis (UC) and Crohn's disease (CD). There are a large number and variety of intestinal bacteria in the human intestinal tract. These bacteria maintain a balance with the human environment and participate in the normal physiological processes of the human body. They play a unique role in defending against pathogen invasion, maintaining the homeostasis of the human immune system and metabolizing substances. Intestinal flora imbalance may be one of the pathogenic factors of IBD, and restoring the disturbed intestinal flora has become a research hotspot in the prevention and treatment of IBD. Changyanning is mainly composed of Dijincao grass, yellow hairy ear grass, camphor tree roots, maple leaves, and so on. Clinical studies have shown that Changyanning alone or in combination has a significant effect on ulcerative colitis, but the treatment mechanism is not yet clear. In this study, we established an IBD animal model to explore the therapeutic mechanism of Changyanning on inflammatory bowel disease and its effect on intestinal flora. *Research Methods*. Male C57BL/6 SPF mice were given free access to 4% dextran sulfate sodium (DSS) solution for 7 days to establish an ulcerative colitis model. After the model was established, different doses of Changyanning tablets, Changyanning granules, and sulfasalazine were given by gavage for 7 days. The relieving effects of the above drugs on the symptoms of inflammatory bowel disease were evaluated by evaluating the mouse/rat body weight, survival rate, disease activity index, colon length, pathological tissue score, and other indicators. *Results*. The DSS-induced IBD mouse model showed significant increases in weight loss, DAI score, and pathological score. Both Changyanning tablets and granules can relieve the weight loss of mice, restore the colon length, and protect the colon tissue structure of mice. In reducing DAI and pathological scores in mice, Changyanning granules had a better effect. In conclusion, Changyanning can significantly improve the quality of life of IBD model animals, relieve intestinal inflammatory response, and relieve colonic edema, ulceration, and necrosis. The results show that Changyanning has a certain therapeutic effect on IBD. This study also provides experimental evidence for the application of Changyanning in the treatment of IBD, which is of great significance to its clinical application. The trail is registered in ChiCTR with number (TRN) ChiCTR2000028830.

## 1. Introduction

Intestinal flora is a huge population of bacteria that live in the human gut. The intestinal flora plays a huge role in the human body's material metabolism and immune regulation and is an inseparable part of the human body. Therefore, the intestinal flora can be regarded as another major organ of the human body. With the development of gut microbial genomics, more and more attention has been paid to the study of gut microbiota. The composition and function of the gut microbiota and its causal relationship with some diseases are becoming clearer. The gut microbiota holds great promise in the treatment of many diseases. Inflammatory bowel diseases include Crohn's disease and ulcerative colitis, which are characterized by chronic inflammation of the intestinal mucosa. IBD has now become a global healthcare problem, and its incidence is on the rise globally. From 1920 to 2010, the average annual incidence of Crohn's disease increased from 1.2 percent to 23.3 percent, and the average annual incidence of ulcerative colitis increased from 2.4 percent to 18.1 percent [1–3]. Incidence rates continue to rise in South America, Eastern Europe, Asia, and Africa [4, 5]. The difference between CD and UC is mainly manifested in terms of pathophysiology and clinical manifestations [4]. The symptoms of UC mainly include abdominal pain, diarrhea, mucus, pus and blood in the stool, and extraintestinal symptoms. In addition, UC may present with nonspecific symptoms such as fever, loss of appetite and weight, fatigue, and primary amenorrhea [6]. The main manifestations of CD are abdominal pain, diarrhea, and abdominal mass, with fistula formation and perianal abscess lesions seen in patients. It is characterized by segmental accumulation of chronic non-granulomatous inflammation of the full thickness of the bowel, with fissured ulcers and a cobblestone-like appearance in the lesioned mucosa, affecting the terminal ileum and perianal region [7, 8]. The pathogenesis of IBD is still not fully understood. Genetic factors and external factors such as irregular diet, long-term antibiotic use, or long-term mental stress are all related to the occurrence of IBD [9]. The main treatment of IBD is drug therapy, which is mainly used to induce or maintain remission of symptoms, and there is no complete cure yet. The main clinical treatment drugs for IBD are salicylic acid, glucocorticoid, and immunosuppressant. Salicylic acids can exert anti-inflammatory effects by reducing the release of proinflammatory factors in the intestine and are often used clinically in patients with mild to moderate symptoms of enteritis. However, salicylic acid drugs have more serious adverse reactions such as gastrointestinal tract, and it has also been reported that patients can experience kidney damage after taking them [10]. Glucocorticoids can relieve inflammation by inhibiting the release of proinflammatory substances and are commonly used clinically in patients with moderate to severe symptoms of enteritis. However, long-term or large doses are prone to drug resistance and a variety of adverse reactions [11]. Immunosuppressive drugs can inhibit the proliferation of inflammatory cells and are mainly used to induce remission or maintain remission of hormone-dependent Crohn's disease that is difficult to treat clinically. However, patients are prone to adverse reactions such as nausea, vomiting, and diarrhea after taking them [12]. In conclusion, although salicylic acid drugs, hormone drugs, or immunosuppressive drugs can alleviate the clinical symptoms of IBD, there are shortcomings such as easy relapse after drug withdrawal and low compliance of patients with long-term use.

Due to urbanization and rapid industrialization, the traditional way of life has changed dramatically. Lifestyle changes have led to an increase in the incidence of IDB, and people have begun to explore the pathogenesis of IBD [13]. However, the pathogenesis of IBD is not yet clear, and the main influencing factors include genetics, environment, intestinal microecology, and immunity. More than 230 genetic genes have been identified to be associated with an increased risk of IBD. Most IBD susceptibility genes are associated with pathways involved in immune-microbe interactions, including microbial detection and immune activation and suppression. Some of these genes encode proteins involved in bacterial recognition, including interleukin IL-23, IL-10 receptor, and ATG16-1 [14]. The prevalence of IBD around the world over the past 30 years suggests that a single genetic mutation is not the only cause of the disease [15]. It has been reported that a large number of bacteria, fungi, and bacteriophages are present in the gut; the gut microbiome is 10 times the number of human cells; and the associated genetic material is 100 times more [16]. Interactions between the gut microbiome and the mucosal immune system have been identified as key to contributing to chronic inflammation. At the same time, alterations in gut microbiome diversity and composition may play a key role in the pathogenesis of IBD. Since the discovery that the microbiota plays a key role in inflammatory bowel disease, there have been an increasing number of studies on the efficacy of fecal microbiota transplantation in intestinal and extraintestinal diseases, and changes in the gut microbiota in IBD have attracted widespread attention.

A large number of studies have shown that targeting intestinal flora as the therapeutic target of IBD has a good effect. For example, *Bifidobacterium*, Collinsella, *Lachnospira*, and Roseburia are related to the effectiveness of TNF-*α* inhibitors in the treatment of CD. The normal intestinal flora is involved in regulating the host's immune response and preventing pathogenic substances from invading the human body, so it is also called the second largest immune system in the human body. When the intestinal flora is disturbed, the microbial barrier function is damaged, leading to the invasion of pathogenic microorganisms and the production of inflammation. In recent years, supplementation of probiotics (such as *Lactobacillus* and *Bifidobacterium*), fecal bacteria transplantation, and traditional Chinese medicine intervention have achieved good results in the treatment of IBD and can effectively relieve its clinical symptoms.

## 2. Related Work

### 2.1. Gut Flora

Microecological studies have shown that the normal human intestinal flora is composed of bacteria belonging to 30 genera and 500 species, and the number is extremely large, which can exceed 1014. Most of the bacteria in the gut belong to 5 phyla, namely, Bacteroidetes, Firmicutes, *Actinobacteria*, Proteobacteria, and Verrucomicrobia. Among them, Bacteroidetes and Firmicutes are more abundant, accounting for more than 90% of intestinal bacteria in healthy people, while *Actinobacteria*, Proteobacteria, and Verrucomicrobia are less abundant [17], as given in Table 1. Normal human intestinal flora can be divided into aerobic bacteria, facultative anaerobic bacteria, and anaerobic bacteria, among which obligate anaerobic bacteria have the largest number, accounting for 99.9% of the intestinal flora [18], as given in Table 2. *Bifidobacterium*, *Eubacterium*, *Bacteroides*, *Peptococcus*, and so on account for a large number of several types of bacteria. Others such as *Escherichia coli*, *Enterococcus*, *Lactobacillus*, and *Veillonella* account for a small number. Although the types of gut bacteria are roughly the same, the specific composition and proportion of gut microbiota vary greatly between individuals and at different stages of each individual.

With the growth, development, and aging of people, the intestinal flora is also undergoing continuous succession. Babies are born with a sterile gut, and after birth, bacteria can invade and colonize the body through the mouth and anus. Because the intestinal environment of newborns is in an aerobic state, the bacteria that appear early are aerobic bacteria, such as *Enterococcus* and *Escherichia coli*. After 2 days of birth, anaerobic bacteria such as *Bifidobacterium* colonize and grow rapidly, gradually replacing aerobic bacteria as dominant bacteria, and the intestinal flora gradually stabilizes after 3 months. Studies have shown that the intestinal flora of infants is close to the level of adult intestinal flora at the age of 2–3 [19]. As people age, the intestinal flora will also undergo a certain degree of succession; that is, the number of anaerobic bacteria such as *Bacteroides* and *Bifidobacterium* decreases and the number of Firmicutes increases. The gut microbiota maintains a certain stable state in a certain period of time, but it is not static, and it will be affected by various reasons, such as changes in dietary structure, environmental factors, and disease states. Some studies have found that after changing people's dietary structure, the intestinal flora changes significantly within a period of time (within 24 hours). Different environments can also affect the intestinal flora, such as the change of seasons and the height of altitude.

### 2.2. Gut Microbiota and IBD

Under normal circumstances, the intestinal flora and the human body maintain a certain balance and participate in human life activities together. When various reasons break this balance, such as flora shift, immune disorder, and flora imbalance, the intestinal flora may be stored in some diseases. Studies have shown that the occurrence of IBD is closely related to the intestinal flora, which is mainly reflected in the following aspects. (1) Sterility and no inflammation are manifested in the immunodeficient IBD animal model obtained by gene knockout, setting a sterile intestinal environment. It will not induce the occurrence of IDB. (2) During the treatment of some IBD patients, the application of antibiotics against the intestinal flora has a certain effect. A number of studies [20–22] have found that IBD patients have intestinal flora imbalance, which is mainly reflected in two aspects: one is the increase in the number of pathogenic bacteria, and the other is the change in the normal proportion of intestinal flora. Ormsby [20] and others analyzed the discriminative specimens of CD patients and found that the content of intestinal bacteria was significantly higher than that of normal people. Wang [21] et al. quantitatively analyzed the intestinal flora of CD patients and found that the content of butyrate-producing bacteria in the intestines was significantly lower than that of normal people. Zhang [22] and others conducted a statistical study on more than 120 CD patients and found that the number of *Escherichia coli* and *Enterococcus* spp. in patients with active CD was higher than that of normal people, while the number of probiotics such as *Bifidobacterium* and *Lactobacillus* decreased. Some researchers found that the number of probiotics such as *Bifidobacterium*, *Bacteroides*, and *Lactobacillus* increased in CD patients. The reason may be the result that the intestinal flora plays a role in regulating the intestinal flora through the intestinal mucosal barrier after the intestinal flora is disturbed. The increase of pathogenic bacteria and the imbalance of intestinal flora can induce and promote the occurrence and development of IBD in the following ways. (1) The number of intestinal pathogenic bacteria increases. Pathogenic bacteria destroy the normal intestinal mechanical barrier and immune barrier through invasive force and secreted toxins, increase the permeability of intestinal mucosa, and create conditions for bacterial translocation. The translocated bacteria overactivate the immune response, causing intestinal tissue to be attacked and damaged by the immune system. (2) Dysbiosis in the gut leads to a decrease in the number of normally existing probiotics. Normally existing intestinal probiotics such as bifidobacteria and lactobacilli can inhibit the growth of pathogenic bacteria through various effects. (3) The imbalance of intestinal flora breaks the normal state of immune tolerance of the body.

In general, the pathogenesis of IBD induced by intestinal flora imbalance can be summarized as follows: in individuals with genetic susceptibility factors, genetic, environmental, and pathogenic bacteria increase; immune tolerance is broken; and immune overactivation is a combination of factors. Under the action, the pathological process of IBD is induced.

Animal models of IBD include genetically engineered models as well as chemically induced models. Among them, genetic engineering models include transgenic or gene-targeted mouse strains, adoptive T cell transfer, and spontaneous models of IBD. Disadvantages of this type of model are developmental abnormalities caused by genetic defects that arise in genetic engineering, or high individual differences between the permeability and activity of colitis. The chemical-induced model of intestinal inflammation has the advantages of rapid induction and relatively simple operation and is the most commonly used animal model of IBD, such as DSS (dextran sulfate sodium salt), TNBS (trinitrobenzene sulfonic acid), oxazolone, and other induced models. These models allow experiments in immunocompetent mice, avoiding some of the disadvantages of genetically engineered colitis models. DSS is a water-soluble sulfated polysaccharide with a molecular weight between 5 and 1400 kDa. Adding 40–50 kDa DSS to drinking water can induce mice to form the most human-like UC model, which is typically characterized by weight loss, bloody diarrhea, ulcers, and epithelial cell loss and neutrophil infiltration. This model is fast, simple, and reproducible and can be used to establish acute, chronic, and recurrent models of intestinal inflammation by adjusting the concentration and administration frequency of DSS, so it is widely used in IBD research. This model has been used to study the effects of the gut microbiome and induced compositional changes, such as dietary factors, on the development of colitis. Our purpose was to study the therapeutic effect of Changyanning tablets and granules on acute colitis mice and to clarify their mechanism of action. Therefore, in this paper, mice were allowed to freely drink 4% DSS solution to establish an acute IBD model and conduct subsequent experiments.

### 2.3. General Situation of Research on Changyanning

Changyanning mainly contains Chinese herbal medicines such as Dijincao, Huang Mao Er grass, camphor tree root, Elsholtzia ciliata and maple leaves. Dijincao is commonly used in traditional Chinese medicine for jaundice, dysentery, and enteritis. The components contained in it have anti-inflammatory, antioxidant, antifungal, anti-hepatitis B virus, and other pharmacological activities and have been proved to have anti-invasive effects against early breast cancer and transfer. It has the functions of clearing away heat and removing dampness, detoxification, and swelling and is often used in traditional Chinese medicine for the treatment of cholestasis, hepatitis, enteritis, and other diseases. Maple leaves dispel wind and dampness are mainly used to treat dysentery, enteritis, and other diseases. At present, Changyanning is mainly used alone or in combination with other drugs for the treatment of ulcerative colitis, acute enteritis, and acute infectious diarrhea. It is also used for the treatment of acute bacterial dysentery, viral enteritis, and acute diarrhea in children. Studies have shown that Changyanning has the effect of treating chronic ulcerative colitis and enhancing cellular immune function, which can improve the symptoms of simple adhesive intestinal obstruction in mice to a certain extent and has the effect of enhancing intestinal peristalsis and repairing intestinal barrier damage.

Although some studies have shown the effectiveness of Changyanning in combination with other drugs in the treatment of inflammatory bowel disease, the specific mechanism of Changyanning in the treatment of inflammatory bowel disease is still unclear. Therefore, this study explored its therapeutic mechanism, including its effect on the intestinal flora of IBD.

## 3. The Therapeutic Effect of Changyanning on DSS-Induced IBD in Mice and the Regulation of Intestinal Flora

### 3.1. The Design Idea of This Experiment

In this paper, the mechanism of the classic prescription Changyanning in the treatment of inflammatory bowel disease and its effect on the intestinal flora of the IBD model were investigated. The content of the study is as follows:

1. DSS-induced mice were used to establish an IBD animal model.
2. The therapeutic effects of Changyanning tablets and granules on IBD model were evaluated from the aspects of disease activity index, colon length change, and pathological score.
3. High-throughput sequencing was performed on the feces of mice/rats in each group to compare the diversity and composition of intestinal flora. The technical roadmap of this experiment is shown in Figure 1.

### 3.2. Experimental Materials

The instruments used in this experiment are given in Table 3.

### 3.3. Methods

#### 3.3.1. Experimental Drug Configuration

4% DSS: A 4% DSS solution was prepared with double-distilled water.

Sulfasalazine: we accurately weighed 1 g of SASP and added it to 50 ml of double-distilled water to dissolve it to a final concentration of 20 mg/mL.

Changyanning tablets: after Changyanning was ground into powder with a mortar, 3.75 g, 7.5 g, and 15 g were weighed, and 50 mL of double-distilled water was added to prepare the suspension solutions of the three dose groups of Changyanning tablets: low (0.075 g/mL), medium (0.15 g/mL), and high (0.3 g/mL).

Changyanning granules: we weighed 5 g, 10 g, and 20 g of Changyanning granules, respectively, and added 50 mL of double-distilled water, respectively, to prepare the solutions of three dose groups of Changyanning granules: low, medium, and high, with concentrations of 0.1 g/mL, 0.2 g/mL, and 0.4 g/mL.

#### 3.3.2. DSS-Induced Acute Colitis Model in Mice

72 male C57BL/6 SPF mice were randomly divided into 9 groups according to body weight after one week of adaptive feeding in a temperature of 18–23 degrees Celsius and a 12-hour light/dark cycle, as given in Table 4. The mice in each group (except the control) were allowed to freely drink the 4% DSS solution prepared with double-distilled water for 7 days at 6 mL/mouse/day (the DSS solution was replaced every 2 days) to induce the mouse model of inflammatory bowel disease. At the same time of establishing the model, the corresponding drugs were administered by intragastric administration at the same time twice a day according to the administration volume of 0.1 mL/10 g for 7 days. The control and DSS groups were given a therapeutic drug solvent (physiological saline), the mice were sacrificed by cervical dislocation on the 8th day, and the mice were dissected for sampling.

#### 3.3.3. Disease Activity Index Score and Colon Length Assessment

The disease activity index is a common index for evaluating colonic injury models in experimental animals and can be used to evaluate the symptoms of weight loss, diarrhea, and blood in the stool in mice treated with DSS. Therefore, we need to record the body weight, activity status, fecal characteristics, and blood in the stool of the mice every day.  Table 5 provides the defecation conditions and stool characteristics of the mice in each group. On the 8th day of the experiment, after the colon was dissected, the colon was observed for edema, adhesion, ulcer, necrosis, and other pathological changes, and the length of the colon was measured with a ruler and photographed for recording. According to the above two indicators, the efficacy of the drug on UC was preliminarily judged.

#### 3.3.4. Colon Tissue Paraffin Section and HE Staining

For colon sampling, after the experiment, the mice were sacrificed by cervical dislocation; the colon tissue was immediately dissected; and the length of the colon was measured and photographed for comparison. After collecting part of the feces in the colon, the colon tissue was washed with normal saline, and a part of the colon tissue was placed in a labeled cryovial, frozen in liquid nitrogen, and then transferred to a −80°C refrigerator for storage. The remaining colon tissue was placed in a 15 mL centrifuge tube containing 10% paraformaldehyde for overnight fixation for HE staining.

#### 3.3.5. Histopathological Scoring and Resolving Samples for DNA Extraction

The scoring criteria refer to the evaluation of the inflammatory state of colon tissue by Sann et al. [23]. We used the sum of the scores for “progression of inflammation,” “inflammation cell infiltration,” “crypt damage,” “crypt abscess,” “submucosa edema,” “goblet cell loss,” and “reactive epithelial cell hyperplasia” as the HS and identified the differences in HS among the groups. Total DNA from 64 mouse fecal samples was isolated and extracted using the Stool DNA Kit, and the 16S rRNA variable region (V3 + V4) was amplified by PCR using the primers given in Table 6. PCR amplification products were detected by 2% agarose gel electrophoresis, and target fragments were recovered by AxyPrep PCR Cleanup Kit. The purified PCR products were quantified on the Qubit fluorescence quantitative system using the Quant-iT PicoGreen dsDNA Assay Kit.

#### 3.3.6. Data Statistical Processing and Analysis

The gut microbiota was analyzed using FLASH 1.2.8 software for splicing sequences, VSEARCH 2.3.4 software for filtering chimeras and OTU clustering, QIIME 1.8.0 software for *α* and *β* diversity analysis, and R 3.4.4 language mapping software. Statistical analysis of other data was carried out using SPSS 22.0 software. One-way analysis of variance was used to compare the differences between groups, and Dunnett's method was used for comparison between groups.

## 4. Experimental Results and Discussion

### 4.1. Effects of Changyanning on the General State of DSS-Induced IBD Model Mice

During the continuous administration period, the mice in the normal group grew well, and their body weight increased slowly. The body weight of the DSS group and each drug intervention group decreased, and with that of the DSS group decreasing the most and the fastest. Compared with that of the DSS group, the weight of the mice in each drug intervention group partially recovered or slowed down. During the administration period (days 2–8), the mice given Changyanning tablets or granules were observed to have less weight loss on the 2nd and 3rd days than the DSS group, but on the 8th day, each administration group was significantly different from the DSS group. Weight loss in the DSS group was comparable, about 25%. The analysis of mouse survival rate is given in Table 7. It can be seen from Table 7 that the survival rate of various mice is ≥75%. Dead mice were present in most groups. The survival rate of the Changyanning tablet group was higher than that of the Changyanning granule group, and there were no dead mice in the CYN Tab.M and CYN Tab.H groups.

During the experiment, it was observed that the mice in the DSS group had severe diarrhea and bloody stools, and the mice in the drug intervention group had occasional bloody stools. The experimental results showed that the DAI score of the DSS group was significantly higher than that of the normal group (*P* < 0.0001 vs. control). After drug intervention, the DAI scores of each group were decreased, among which Changyanning granule low-dose and high-dose group and Changyanning tablet group had significant effects (*P* < 0.01 vs. DSS), but there was no obvious dose-dependent effect. The disease activity index scores of mice in each group on the 8th day of administration of Changyanning tablets and Changyanning granules are shown in Figure 2. DSS-induced mice have significant disease responses. SASP, Changyanning tablets, and Changyanning granules can all reduce the weight loss rate of UC mice in the early stage of DSS-induced inflammatory bowel disease to a certain extent, improve the growth status and macroscopic disease symptoms of mice, and have an anti-UC effect, especially in the high-dose group of particles (4 g/kg).

### 4.2. Protective Effect of Changyanning on Colon Tissue Structure in DSS-Induced IBD Model Mice

After drug treatment, the colonic condition of mice in Changyanning tablet and granule group and SASP group improved compared with DSS group. In the Changyanning tablet and granule group, the intestinal wall structure was clear, the shape was normal, the gland crypts were relatively neatly arranged, the goblet cells were increased, the inflammatory cell infiltration was improved, and the reactive epithelial cells were neatly arranged. Colonic HS was significantly decreased in CYN Tab.H mice (*P* < 0.01 vs. DSS). Compared with the histopathological scores of the DSS group, those of the mice in each group treated with Changyanning granules decreased to a certain extent; those of the high-dose group decreased significantly (*P* < 0.001 vs. DSS), followed by the low-dose group (*P* < 0.01 vs. DSS); and there was no statistical significance in the middle-dose group. The detailed results are given in Table 8. The inflammatory infiltration was slightly improved in the SASP group, but goblet cells were lost, epithelial cells proliferated, and only a few crypt shapes and goblet cells were observed. Compared with the DSS group, the SASP group had decreasing HS score, but there was no significant difference.

In conclusion, DSS induces inflammatory lesions of colon tissue in mice, and Changyanning tablets and granules can effectively improve colon damage and inflammatory response and further relieve acute colitis caused by DSS, with a better effect than that of SASP, especially Changyanning tablets (high doses of Changyanning granules).

### 4.3. Discussion

Changyanning granules have a significant effect on the treatment of ulcerative colitis in mice caused by DSS. The improvement effect is better in the disease state of the model mice and the pathological state of the colon, and the results can provide reference value and experimental basis for its clinical application. Changyanning tablets can significantly improve various disease states of ulcerative colitis in mice caused by DSS, reduce the mortality rate of mice, and improve the overall state of mice such as activity and hair. However, there was no statistical difference in the direct improvement effect on colon tissue, which may be related to the characteristics of traditional Chinese medicine prescriptions in improving the overall state of the body.

## Figures and Tables

**Figure 1:** Experimental technology roadmap.

**Figure 2:** Disease activity index scores of mice in each group on the 8th day of administration of Changyanning tablets and Changyanning granules.

**Table 1:** The main types of intestinal flora in the human body.

Phylum	Genus	Number
Bacteroidetes	*Bacteroides*, *Porphyromonas*, and *Puccinia*	More, accounting for more than 90%
Firmicutes	*Clostridium*, *Clostridium* Tenella, *Eubacterium*, *Ruminococcus*, and *Lactobacillus*	
*Actinobacteria*	*Bifidobacterium* and gas-producing Collinsella	
Proteobacteria	Enterobacteriaceae bacteria, *Helicobacter pylori*	Less quantity
Verrucomicrobia	*Verrucomicrobium*	

**Table 2:** Number of common bacteria in feces.

Type	Flora	Number (/g feces)
Beneficial bacteria	*Bifidobacterium*	10^8^–10^12^
	*Lactobacillus*	10^8^–10^10^

Opportunistic pathogen	*Enterococcus*	10^6^–10^10^
	*Enterobacter*	10^4^–10^10^
	*Bacteroides*	10^6^–10^10^

Pathogenic bacteria	*Pseudomonas aeruginosa*	10^4^
	*Staphylococcus*	10^4^–10^7^

**Table 3:** Experiment apparatus.

Main instruments and models	Manufacturer
Embedding machine	German Company Leica
Tablet machine	German Company Leica
Sheet oven	German Company Leica
Dehydrator (ASP300)	German Company Leica
Slicer (RM2235)	German Company Leica
Inverted microscope	Olympus Life Science
Electronic balance (YP10002)	Shanghai Guangzheng Medical Instrument Co., Ltd.
Electronic balance (AG204)	Mettler Toledo
Electric thermostatic water tank (DK-8D)	Shanghai Jinghong Experimental Equipment Co., Ltd.
Benchtop refrigerated centrifuge (5417R)	Eppendorf
Microplate reader (ELX808)	BioTek
Biological sample grinder	Bertin Technologies

**Table 4:** Grouping and dosing.

Group	Number	Medicine	Dosage
Control	8	Normal saline	0
DSS	8	Normal saline	0
SASP	8	SASP	200 mg/kg
CYN Tab.L	8	Changyanning tablets	0.75 g/kg
CYN Tab.M	8	Changyanning tablets	1.5 g/kg
CYN Tab.H	8	Changyanning tablets	3 g/kg
CYN Gra.L	8	Changyanning granules	1 g/kg
CYN Gra.M	8	Changyanning granules	2 g/kg
CYN Gra.H	8	Changyanning granules	4 g/kg

**Table 5:** DAI scoring method.

Score	Weight loss (%)	Stool traits	Fecal occult blood/colon bleeding
0	0	Normal stool, in a ball shape	No colon bleeding or blood in the stool
1	1–5	Soft, mushy stools that do not stick to the anus	Fecal occult blood or minor bleeding spots in the colon
2	5–10	Moderate diarrhea, uneven stools, sticky anus	Bloody stools or visible bleeding in the colon
3	10–15	Diarrhea, watery stools	Fresh bleeding
4	>15	—	—

**Table 6:** Primer selection for bacterial 16S rRNA gene sequencing.

Sequencing region	Primer name	Primer sequence
515F-805R	515F	5′-GTGYCAGCMGCCGGTAA-3′
	805R	5′-GGACTACHVGGGTWTCTAAT-3′

**Table 7:** Mouse survival statistics.

Group	Survival number	Number of deaths	Survival rate (%)
Control	8	0	100
DSS	7	1	87.5
SASP	7	1	87.5
CYN Tab.L (0.75 g/kg)	6	2	75
CYN Tab.M (1.5 g/kg)	8	0	100
CYN Tab.H (3 g/kg)	8	0	100
CYN Gra.L (1 g/kg)	7	1	87.5
CYN Gra.M (2 g/kg)	6	2	75
CYN Gra.H (4 g/kg)	7	1	87.5

**Table 8:** Mouse colon histopathology score (mean ± SD).

Group	Number	Pathological score
Control	8	1.635 ± 1.24
DSS	7	10.58 ± 2.23^*∗∗∗∗*^
SASP	7	7.89 ± 3.15
CYN Tab.L (0.75 g/kg)	6	9.07 ± 2.17
CYN Tab.M (1.5 g/kg)	8	9.15 ± 2.91
CYN Tab.H (3 g/kg)	8	6.26 ± 1.12^*∗∗*^
CYN Gra.L (1 g/kg)	7	6.78 ± 2.14^*∗∗*^
CYN Gra.M (2 g/kg)	6	7.86 ± 1.18
CYN Gra.H (4 g/kg)	7	5.76 ± 1.52^*∗∗∗*^

Note. ^*∗∗∗∗*^*P* < 0.0001 vs. control; ^*∗∗*^*P* < 0.01 vs. DSS; ^*∗∗∗*^*P* < 0.001 vs. DSS.

## Data Availability

The data used to support the findings of this study are available from the corresponding author upon request.
